# Changes of Radial Diffusivity and Fractional Anisotopy in the Optic Nerve and Optic Radiation of Glaucoma Patients

**DOI:** 10.1100/2012/849632

**Published:** 2012-04-19

**Authors:** Tobias Engelhorn, Georg Michelson, Simone Waerntges, Marlen Otto, Ahmed El-Rafei, Tobias Struffert, Arnd Doerfler

**Affiliations:** ^1^Department of Neuroradiology, University of Erlangen-Nuremberg, Schwabachanlage 6, 91054 Erlangen, Germany; ^2^Department of Ophthalmology, University of Erlangen-Nuremberg, Schwabachanlage 6, 91054 Erlangen, Germany; ^3^Department of Computer Science, University of Erlangen-Nuremberg, Martensstrasse 3, 91058 Erlangen, Germany

## Abstract

Purpose of this study was to evaluate with diffusion-tensor imaging (DTI) changes of radial diffusivity (RD) and fractional anisotropy (FA) in the optic nerve (ON) and optic radiation (OR) in glaucoma and to determine whether changes in RD and FA correlate with disease severity. Therefore, glaucoma patients and controls were examined using 3T. Regions of interest were positioned on RD and FA maps, and mean values were calculated for ON and OR and correlated with optic nerve atrophy and reduced spatial-temporal contrast sensitivity (STCS) of the retina. We found, that RD in glaucoma patients was significantly higher in the ON (0.74 ± 0.21 versus 0.58 ± 0.17·10^−3^ mm^2^ s^−1^; *P* < 0.05) and OR (0.79 ± 0.23 versus 0.62 ± 0.14·10^−3^ mm^2^ s^−1^; *P* < 0.05) compared to controls. Aside, FA was significantly decreased (0.48 ± 0.15 versus 0.66 ± 0.12 and 0.50 ± 0.20 versus 0.66 ± 0.11; *P* < 0.05). Hereby, correlation between changes in RD/FA and optic nerve atrophy/STCS was observed (*r* > 0.77). In conclusion, DTI at 3 Tesla allows robust RD and FA measurements in the ON and OR. Hereby, the extent of RD increase and FA decrease in glaucoma correlate with established ophthalmological examinations.

## 1. Introduction

Glaucoma is responsible for approximately 10% of the cases of blindness throughout the world and thus is the third leading cause of blindness with more than 8 million cases each year [1]. Glaucoma is considered a nervous-system-based degenerative disease that is only partially influenced by ocular factors [2]. Moreover, neuronal degeneration involving all parts of the central visual pathways was documented at autopsy in a patient who had advanced open-angle glaucoma and severe visual field losses in both eyes [3].

Central neuronal degeneration can be assessed noninvasively using diffusion tensor imaging (DTI) with calculation of radial diffusivity (RD) and fractional anisotropy (FA). The parameter fractional anisotropy (FA) measures the orientation coherence of diffusion and provides information about the fiber integrity. The radial diffusivity (RD) is the apparent water diffusion coefficient in the direction perpendicular to the axonal fibers. It represents a parameter of demyelination or glia cell impairment [4].

Hence, goal of this study was to evaluate whether 3 Tesla DTI with calculation of RD and FA in different sections of the visual pathways can assess the spread of glaucomateous damage within the central nervous system and to determine whether these functional MRI-derived parameters correlate with disease severity in 22 severely ill patients with glaucoma aged 37 to 86 years and 20 age-matched control subjects aged 45 to 83 years.

## 2. Materials and Methods

The study was conducted in accordance with the Declaration of Helsinki on Biomedical Research Involving Human Subjects. The institutional Clinical Investigation Ethics Committee approved the study protocol, and written informed consent was obtained from all subjects prior to the study after explanation of the nature and possible consequences of the study.

Eyes were assessed in full ophthalmologic examinations. Available additional examinations were referred to for evaluation, including Heidelberg Retinal Tomography (Heidelberg Engineering, Heidelberg, Germany), automated perimetry (Octopus 101 dG2; Interzeag, Schlieren, Switzerland), spatial-temporal contrast sensitivity (STCS, frequency doubling test; Carl Zeiss Meditec AG, Jena, Germany), nonmydriatic fundus images (nonmyd-alpha 45; Kowa Optimed, Inc, Torrance, CA), and measurement of intraocular pressure.

MRI was performed on a 3T high-field scanner (Magnetom Tim Trio, Siemens Healthcare AG, Erlangen, Germany) with gradient field strength up to 45 mT/m (72 mT/m effective). The anatomical data were obtained in a T1-weighted 3D-MPRAGE sequence (TR = 900 ms, TE = 3 ms, FoV = 23 × 23 cm, acquisition matrix size = 512 × 256 reconstructed to 512 × 512, reconstructed axial plans with 1.2 mm slice thickness). DTI was performed in the axial plane with 4 mm slice thickness using a single-shot, spin echo, echo planar imaging (EPI) diffusion tensor sequence thus covering the whole visual pathway (TR = 3400 ms, TE = 93 ms, FoV = 23 × 23 cm, acquisition matrix size = 256 × 256 reconstructed to 512 × 512, number of signal averages = 7, partial Fourier acquisition = 60%). Diffusion weighting with a maximal *b*-factor of 1000 s/mm^2^ was carried out along 15 icosahedral directions complemented by one scan with *b* = 0. Datasets were automatically corrected for imaging distorsions and coregistered in reference to T1-weighted MPRAGE images.

DTI data were interpolated in the Log-Euclidean framework to avoid the swelling effect. Then, the data were further processed and the estimated segmented optic radiation was checked for concordance with anatomical knowledge. The slice, which soonest included the lateral geniculate nucleus (LGN), was chosen for further proceeding and calculations. Analysis of the segmentation errors showed that additionally, anatomical structures were segmented, which are not belonging to the optic radiation. These structures were manually removed. Predominantly, parts of the optic tract, the forceps major of the corpus callosum, which proceeds medial of the optic radiations and all tracts, which do not connect to the visual cortex were concerned. The special anatomy in the area of the LGN has to be considered in more detail. In axial slices of this region the axons of the optic radiation, which derive from the LGN, overlap with the distal part of the optic tract, which connects to the LGN. Exclusion of this area would effectuate a loss of information from the LGN and origin of the optic radiation. An inclusion would produce acquisition of the distal part of the optic tract. As we decided in favour of the latter solution, some information from the distal part of the optic tract was included in our calculations of the mean values of the radial diffusivity (RD) and fractional anisotropy (FA).

These and further calculations such as determining the independent elements of the diffusion tensor, deriving the corresponding eigenvalues and eigenvectors, and calculation of RD and FA maps were performed with a dedicated software package (Neuro 3D, Siemens Healthcare AG, Erlangen, Germany). Drawing the regions of interest (ROIs) of approximately 9 mm^2^ on the RD and FA maps superimposed over the T1-weighted 3D-MPRAGE sequence was done by two experienced neuroradiologists (T. S. and A. D.), who were blinded to the patients' clinical data. The following ipsi- and contralateral ROIs were used for evaluation of RD and FA:

  ROI 1: the intracranial part of the ON directly before the optic chiasm (Figure 1(b));
  ROI 2: the optic radiation (OR) directly after the lateral geniculate nucleus (Figure 1(e));
  ROI 3: the OR on the level of the posterior horn of the lateral ventricle (Figure 1(e));
  ROI 4: the OR directly before its cortical spread (Figure 1(f)).

These ROIs were chosen to examine the 3rd neuron (optic nerve) as well as the 4th neuron (optic radiation) of the visual pathways. Hereby, the intracranial part and not the intraorbital part of the ON was chosen to avoid movement artefacts that affect the intraorbital part caused by eye motion during the MRI examination.

Statistical analyses were performed using the PASW software (release 18.0, SPSS Inc. Chicago, IL, USA).

## 3. Results

The ophthalmological examination revealed no significant affection of the eyes in all 20 controls. Aside, MRI revealed no space occupying lesions or infarction along the extra- and intracranial visual pathway in all 42 test persons.

Measurement of RD and FA in ipsi- and contralateral ROIs was feasible in all test persons. Mean evaluation time was 32 minutes per patient.

Cronbach-*α* at the 95% confidence interval for RD was 0.89 (right side, *F* = 2.54, *P* = 0.19) and 0.86 (left side, *F* = 1.65, *P* = 0.27) while for FA it was 0.99 (right side, *F* = 2.34, *P* = 0.15) and 0.88 (left side, *F* = 1.08, *P* = 0.32). Thus, the correlation coefficients of reliability of the RD and FA measurements done by two neuroradiologists were within a very good range of reliability. Hence, the results of both RD and FA measurements were averaged.

In controls, there was good correlation between an increase in RD of both sides with increasing age (*r* = 0.71). The overall percentage change in RD in control subjects between 45 and 83 years was 15.3 ± 5.0%. This difference was significant (*P* = 0.04). Aside, there was good correlation between a decrease in FA of both sides with increasing age (*r* = 0.78). The overall percentage change in FA in control subjects between 45 and 83 years was 33.7 ± 10.7%. This difference was also significant (*P* = 0.02).

Right and left side RD and FA measurements in controls and glaucoma patients were similar and differed only in small ranges up to five percent (no significant differences in all test persons). Hence, the measurements for both sides were averaged and are displayed in Tables 1 and 2.

In glaucoma patients, good correlation between an increase in RD as well as a decrease in FA measured in the intracranial part of the ON and in the OR and the extent of optic nerve atrophy and STCS of the retina was observed (*r* > 0.77 and *r* > 0.81, resp.).

## 4. Discussion

Physiological changes of white matter tracts in the brain show different regional patterns dependent on age, and circulatory disorders [5–7]. The compromised fiber microstructure may at least in part participate in mechanisms of functional degradation [5]. An anterior-posterior gradient of impairment in the brain was described, which is detectable by diffusion tensor imaging (DTI) [8]. This examination method is based on magnetic resonance imaging (MRI) and characterizes the structure of brain tissue based on underlying water diffusivity [4].

Water diffusion is highly anisotropic in white matter of the nervous system because the overall mobility of the diffusing molecules is limited by intracellular and extracellular compartments, by neurons, glial cells, and by axons [9]. The DTI-derived parameter fractional anisotropy (FA) measures the orientation coherence of diffusion and provides information about the fiber integrity [4, 5], while the radial diffusivity (RD) is the apparent water diffusion coefficient in the direction perpendicular to the axonal fibers. It represents a parameter of demyelination or glia cell impairment [10].

In a recently published study [11], DTI was shown to enable quantitative assessment of the optic radiation by volume rendering of the reconstructed fiber tracts. Hereby, the DTI-derived volume of the optic radiation of glaucoma patients was significantly decreased compared to age-matched controls. To our best knowledge, this is the first study to report qualitative measurements of DTI-derived radial diffusivity (RD) and fractional anisotropy (FA) correlated with established ophthalmological tests in different sections of the 3rd neuron (optic nerve) and 4th neuron (optic radiation) of the visual pathways of glaucoma patients and normal seeing controls using a high-field 3 Tesla MR scanner.

We could demonstrate that (1) measurement of RD and FA in different sections of the visual pathways is feasible, and (2) there is a significant increase in RD as well as a significant decrease in FA in healthy controls with increasing age. (3) Compared to age-matched controls, RD is significantly increased and FA is significantly decreased in the optic nerve and in all examined sections of the optic radiation in glaucoma patients, and (4) there is good correlation between the increase in RD and the decrease in FA and the severity of optic nerve atrophy and retinal impairment quantified with established ophthalmological tests. Thereby, (5) FA is superior to RD in detecting glaucoma-induced intracranial damage.

Hereby, the strong influence of age-related processes on RD and FA is not surprising. Different patterns of RD and FA, suggesting mechanisms of functional degradation, were shown to compromise at least in part the fiber microstructure [5]. Age-related increases in RD as well as decreases in FA, that reflect the axonal integrity including myelination, were seen throughout the brain and several studies [12–14]. In this study, the overall percentage change in RD and FA in control subjects between 45 and 83 years was plus 15.3 ± 5.0 and minus 33.7 ± 10.7%, respectively. As result, RD and FA in different sections of the visual pathways of glaucoma patients were compared to age-matched controls. Hereby, we found a significant change in RD and FA in the optic nerve (3rd neuron of the visual pathways) and in all three sections of the optic radiation (4th neuron of the visual pathways), thus in all sections with a more or less straight axonal direction before the cortical spread.

In contrast, there was no significant change in RD and FA in the intraorbital optic nerve, the optic chiasm, and the lateral geniculate nucleus (RD and FA values not shown). The explanation for this finding is most likely the crossing of axons in the optic chiasm and the reconnection of axons in the lateral geniculate nucleus resulting in a change of the straight axonal direction with subsequent change in RD and FA [15], whereby ineluctably movement of the eyeball subsequently results in movement of the intraorbital optic nerve downgrading the quality of RD and FA assessment in this section of the visual pathways by motion artefacts. This limitation could be overcome with retrobulbar anesthesia or by simply using the intracranial part of the optic nerve as done in this study.

As most important finding, we could demonstrate that there is correlation of MRI-derived changes in RD and FA in the optic nerve and the optic radiation of glaucoma patients with established ophthalmological scores to determine the degree of optic nerve atrophy and reduced spatial-temporal contrast sensitivity of the retina. Hereby, changes in FA with *r* > 0.81 seem to be slightly superior to changes in RD with *r* > 0.77.

In conclusion, there is degeneration of the visual pathways with subsequent characteristic changes in RD and FA along the 3rd and 4th neuron in glaucoma patients. Hereby, the extent of degeneration can be assessed noninvasively by 3 Tesla DTI with robust measurement of RD and FA with correlation to optic nerve atrophy and retinal impairment.

## Figures and Tables

**Figure 1:** Different regions of interest (red circles in the right visual pathways) that were used for evaluation of radial diffusivity (RD) and fractional anisotropy (FA) in glaucoma patients and controls in the left and right visual pathways: intraorbital part of the optic nerve (a), intracranial part of the optic nerve (b), optic chiasm (c), lateral geniculate nucleus (d), and different sections of the optic radiation (e, f). All regions of interest are drawn in a fused dataset of FA-weighted DTI and 3D-MPRAGE sequences (a–c: coronal slides; d–f: axial slides).

**Table 1:** Averaged RD values in different ROI of glaucoma patients and controls.

Localization	Mean RD ± standard deviation (glaucoma patients versus controls)
ROI 1	0.74 ± 0.21 versus 0.58 ± 0.17·10^−3^ mm^2^ s^−1∗^
ROI 2	0.70 ± 0.26 versus 0.55 ± 0.16·10^−3^ mm^2^ s^−1∗^
ROI 3	0.76 ± 0.22 versus 0.60 ± 0.14·10^−3^ mm^2^ s^−1∗^
ROI 4	0.79 ± 0.24 versus 0.65 ± 0.14·10^−3^ mm^2^ s^−1∗^

*Significant lower RD values compared to controls (*P* < 0.05).

**Table 2:** Averaged FA values in different ROIs of glaucoma patients and controls.

Localization	Mean FA ± standard deviation (glaucoma patients versus controls)
ROI 1	0.48 ± 0.15 versus 0.66 ± 0.12*
ROI 2	0.40 ± 0.16 versus 0.57 ± 0.13*
ROI 3	0.48 ± 0.17 versus 0.64 ± 0.11*
ROI 4	0.44 ± 0.22 versus 0.53 ± 0.20*

*Significant lower FA values compared to controls (*P* < 0.05).
